# Glycogen Synthase Kinase 3*β* inhibits BMSCs Chondrogenesis in Inflammation via the Cross-Reaction between NF-*κ*B and *β*-Catenin in the Nucleus

**DOI:** 10.1155/2022/5670403

**Published:** 2022-09-12

**Authors:** Zhenggang Wang, Zhiyi He, Weikai Zhang, Shuang Liang, Kun Chen, Shimeng Xu, Ying Zhang, Peng Cheng

**Affiliations:** ^1^Department of Orthopedics, Tongji Hospital, Tongji Medical College, Huazhong University of Science and Technology, Wuhan 430030, China; ^2^Department of Orthopedics, The First Affiliated Hospital of USTC, Division of Life Sciences and Medicine, University of Science and Technology of China, Hefei 230001, China; ^3^Department of Nephrology, Tongji Hospital, Tongji Medical College, Huazhong University of Science and Technology, Wuhan 430030, China

## Abstract

Inflammation can influence the pluripotency and self-renewal of mesenchymal stem cells (MSCs), thereby altering their cartilage regeneration ability. Sprague-Dawley (SD) rat bone marrow mesenchymal stem cells (BMSCs) were isolated and found to be defective in differentiation potential in the interleukin-1*β-* (IL-1*β*-) induced inflammatory microenvironment. Glycogen synthase kinase-3*β* (GSK-3*β*) is an evolutionarily conserved serine/threonine kinase that plays a role in numerous cellular processes. The role of GSK-3*β* in inflammation may be related to the nuclear factor-*κ*B (NF-*κ*B) signaling pathway and the Wnt/*β*-catenin signaling pathway, whose mechanism remains unclear. In this study, we found that GSK-3*β* can inhibit chondrogenesis of IL-1*β*-impaired BMSCs by disrupting metabolic balance and promoting cell apoptosis. By using the inhibitors LiCl and SN50, we demonstrated that GSK-3*β* regulates the chondrogenesis via the NF-*κ*B and Wnt/*β*-catenin signaling pathways and possibly mediates the cross-reaction between NF-*κ*B and *β*-catenin in the nucleus. Given the molecular mechanisms of GSK-3*β* in chondrogenic differentiation in inflammation, GSK-3*β* is a crucial target for the treatment of inflammation-induced cartilage disease.

## 1. Introduction

Articular cartilage damage is a frequent clinical problem with joint swelling and pain [1]. As the main character of degenerative joint diseases, mainly osteoarthritis and chronic inflammatory joint disease, such as rheumatoid arthritis, it is important to study the mechanism of cartilage damage and how to promote cartilage repair [2, 3]. Bone marrow mesenchymal stem cells (BMSCs) can be induced to differentiate into chondrocytes under certain conditions, therefore they have a potential application in the treatment of cartilage damage, inflammation, and other cartilage diseases [4, 5].

Glycogen synthase kinase-3*β* (GSK-3*β*) is a serine/threonine-protein kinase involved in many intracellular functions [6]. And it is important in regulating the activity of nuclear factor-*κ*B (NF-*κ*B) [7, 8]. The NF-*κ*B signaling pathway plays an essential role in inflammation by regulating the transcription of genes involved in cell growth and cell death. It is reported that NF-*κ*B influences chondrogenic differentiation by down-regulating the mRNA levels of Sox9, a chondrogenic transcription factor [9]. Meanwhile, the expression of NF-*κ*B p65 in growth plate chondrocytes has been shown to facilitate growth plate chondrogenesis [10].

In addition, GSK-3*β* earmarks *β*-catenin for degradation by the proteasome, which mediates the Wnt/*β*-catenin signaling pathway. The Wnt/*β*-catenin signaling pathway widely participates in cellular differentiation, especially in chondrogenesis and osteogenesis [11, 12]. And aberrations in the Wnt/*β*-catenin signaling pathway are often associated with defective cellular differentiation. However, the role of GSK-3*β* in the BMSCs chondrogenesis in IL-1*β*-induced inflammation has not been fully described, and the underling mechanisms deserve exploring.

In this study, we investigated the effect of GSK-3*β* on IL-1*β*-impaired chondrogenesis of BMSCs. Meanwhile, we used LiCl, an inhibitor of GSK-3*β*, to explore the regulation of GSK-3*β* on the NF-*κ*B and Wnt/*β*-catenin signaling pathways. Furthermore, SN50, a specific inhibitor of NF-*κ*B translocation, was used to verify the cross-reaction between NF-*κ*B and *β*-catenin in the nucleus.

## 2. Materials and Methods

### 2.1. Cell Culture and Chondrogenic Differentiation

Sprague-Dawley (SD) male rat BMSCs were purchased from Cyagen Biosciences (RASMX-01001) and were cultured with DMEM/F12 medium (BOSTER, PYG0084) containing 10% fetal bovine serum (Gibico, 10100147) at 37°C with 5% CO_2_ in a humidified incubator. BMSCs were passaged according to the usual method when they were 90% confluent, and the third passage was used in the experiments. Approximately 2.5 × 10^5^ BMSCs were transferred into a 15 mL reaction tube and centrifuged at 150 g for 5 min at room temperature. After incubation in 0.5 mL chondrogenic differentiation medium (CDM; Cyagen Biosciences, RAXMX-90041) at 37°C with 5% CO_2_ for 24 h, the pellets had a round morphology and floated within the medium. Then based on previous researches, the pellets were stimulated with 10 ng/mL IL-1*β* (PeproTech, 211-11B), 10 nM GSK-3*β* (Creative BioMart, 2728R), 10 mM LiCl (Sigma-Aldrich, L9650), and/or 15 *μ*M SN50 (MedChemExpress, HY-P0151) [13–16]. And the CDM was carefully replaced every 2-3 days. After 3 weeks, the pellets were collected and chondrogenic differentiation was evaluated. In addition, BMSCs were seeds at 1 × 10^5^ cells per well in 6-well plates. After incubation for 24 h, the medium was change to the CDM, and BMSCs were stimulated at the same regimen described above. On day 3, BMSCs were harvested to detect apoptosis and explore the mechanisms.

### 2.2. Histological Analysis of Chondrogenic Pellet

The pellets were washed with PBS, fixed with 4% paraformaldehyde for three hours and prepared for paraffin embedding. Then pellets were fixed to a paraffin block and 3 *μ*m sections were obtained using a microtome. For Alcian blue staining, sections were incubated in 1% Alcian blue solution for 30 minutes. For immunofluorescent staining, sections were incubated with 10% donkey serum for 30 min after dewaxing and antigen retrieval. Then sections were incubated with anti-Col 2a antibody (Santa Cruz Biotechnology, sc-52658, 1 : 50) overnight at 4°C. The next day, sections were incubated with FITC conjugated secondary antibody at 37°C for 1 h in the dark. Finally, sections were incubated with 4′,6-diamidino-2-phenylindole (DAPI; Solarbio, C0065) for 5 min and then visualized under a fluorescence microscope (Nikon, Japan).

### 2.3. DMMB Assay of GAG

At the end of the experiment, the conditioned medium was collected, and glycosaminoglycan (GAG) was quantified using a dimethyl-methylene blue (DMMB; Sigma-Aldrich, USA) assay. Briefly, for each well of 96-well plate, 40 *μ*L sample or standard was mixed with 250 *μ*L DMMB solution and incubated at 37°C for 1 h. 525 nm absorption was measured on a microplate ELISA reader. The amount of GAG was calculated by the OD value according to the chondroitin sulfate (Sigma-Aldrich, USA) standard curve.

### 2.4. RNA Extraction and qRT-PCR Analysis

Total RNA was extracted from the pellets using Trizol reagent (Invitrogen, USA) according to the manufacturer's protocol. Reverse transcription was performed using a Superscript III first-strand cDNA synthesis kit (Thermo Fisher Scientific, USA). The expression levels of chondral-related genes Sox9, Collagen 2a, and Aggrecan were assessed by quantitative real-time PCR with SYBR-Green master mix (Thermo Fisher Scientific, USA). GAPDH was selected as an internal control. Gene expression levels were normalized to GAPDH by using the ΔΔCt method. The primers are listed in Table 1.

### 2.5. Western Blotting Analysis

Total proteins were collected from the pellets or BMSCs. And the Nuclear and Cytoplasmic Protein Extraction Kit (Beyotime, P0027) was used to extract proteins from BMSCs. Proteins were separated in 10% SDS-PAGE and transferred to PVDF membranes (Millipore, USA). Then membranes were blocked with 5% BSA for 1 h at room temperature and incubated with primary antibody overnight at 4°C. Specific bands were detected with an HRP-conjugated secondary antibody and were visualized by an enhanced chemiluminescence kit. The expression of protein was normalized to GAPDH (Biotechnology, 60004-1-Ig) or Histone (Abcam, ab179) using Image Lab software (Bio-Rad, USA). For total proteins from the pellets, primary antibodies against Sox9 (CST, 82630), Col 2a, and Aggrecan (Biotechnology, 13880-1-AP) were used. For total proteins from BMSCs, primary antibodies against Bax (CST, 14796), Bcl-2 (Abcam, ab196495), Survivin (CST, 2808), caspase 9 (CST, 9508), cleaved caspase 9 (CST, 9507), caspase 3 (CST, 9662), cleaved caspase 3 (CST, 9661), IKK*β* (CST, 8943), p-IKK*α*/*β*-Ser176/Ser180 (CST, 2697), I*κ*B*α* (CST, 9242), p-I*κ*B*α*-Ser32 (CST, 2859), NF-*κ*B p65 (CST, 8242), p-NF-*κ*B p65 (CST, 3033), *β*-catenin (CST, 8480), p-*β*-catenin (CST, 4176), GSK-3*β* (CST, 12456), and p-GSK-3*β* (CST, 5558) were used. For nuclear and cytoplasmic protein from BMSCs, primary antibodies against NF-*κ*B p65 and *β*-catenin were used.

### 2.6. Apoptosis Evaluation

The apoptotic rate of BMSCs was determined using the flow cytometry (FCM) analysis with an Annexin V-FITC/PI Apoptosis kit (BD Bioscience, USA). BMSCs were harvested and resuspended in a 500 *μ*L binding buffer and stained with 5 *μ*L FITC Annexin V and 5 *μ*L propidium iodide (PI). After incubation for 15 min, the samples were tested using a flow cytometer (BD Bioscience, USA). For each FCM analysis, 10,000 events were recorded. Annexin V+/PI- and Annexin V+/PI+ cells were considered as early and late phase apoptotic cells.

TUNEL staining was performed on BMSCs cultured on 12-well plates using a one-step TUNEL assay Kit (Beyotime, China). According to the manufacturer's instructions, the samples were washed with PBS and fixed with 4% paraformaldehyde for 30 min. Then the samples were incubated with 50 *μ*L of TUNEL detection liquid for 60 min at 37°C in the dark. Finally, nuclei were stained with DAPI and samples were visualized under a fluorescence microscope.

### 2.7. Immunofluorescence

BMSCs were harvested and resuspended in PBS. The suspension was smeared to glass slide and was dried. Cells were fixed with 4% paraformaldehyde, permeabilized in 0.1% TritonX-100, and blocked with 3% BSA. Thereafter, cells were incubated with the primary antibody in blocking buffer against NF-*κ*B p65 and *β*-catenin at 4°C overnight. The next day, cells were incubated with FITC conjugated and TRITC conjugated secondary antibody at 37°C for 1 h in the dark. Finally, cells were stained with DAPI and visualized under a laser confocal microscope (Olympus, Japan).

### 2.8. Statistical Analysis

All experimental group were independently performed in biological triplicate. Data were presented as means ± standard deviation (SD). Statistical analyses were performed using GraphPad Prism 8 (GraphPad Software, USA). Student's *t*-test was used to assess differences between the two groups. One-way ANOVA was used to assess differences among multiple groups. *P* values <0.05 were considered statistically significant.

## 3. Results

### 3.1. Chondrogenic Differentiation of BMSCs in an IL-1*β*-Induced Inflammatory Microenvironment

BMSCs were formed into pellets and cultured in the CDM for 21 days. To establish an inflammatory microenvironment, IL-1*β* was added into the CDM from day 1. The Alcian blue staining intensity of the IL-1*β* group was much lower than those of the control group (Figures 1(a) and 1(b)). And GAG quantity in the conditioned medium also decreased in the IL-1*β* group (Figure 1(c)). Besides, IL-1*β* significantly decreased the expression of Sox9, Collagen 2a (Col 2a), and Aggrecan at both gene and protein levels (Figures 1(d)–1(f)).

### 3.2. GSK-3*β* Disrupts Metabolic Balance of IL-1*β*-Impaired BMSCs

Immunofluorescence staining showed that compared with the IL-1*β* group, the expression of Collagen 2a was decreased in the GSK-3*β*+IL-1*β* group, while was significantly increased in the LiCl+IL-1*β* group (Figure 2(a)). Compared with the control group, GAG quantity in the conditional medium was not changed by GSK-3*β* or LiCl alone, and GSK-3*β* enhanced and IL-1*β*-induced decline in GAG quantity, while LiCl reversed this trend (Figure 2(b)). Accordingly, the expression of Sox9, Col 2a, and Aggrecan were significantly decreased in the GSK-3*β*+IL-1*β* group than in the IL-1*β* group at both gene and protein levels (Figures 2(c)–2(e)).

### 3.3. GSK-3*β* Promotes Apoptosis of IL-1*β*-Impaired BMSCs

Western blotting analysis was used to detect the expression of Bax, Bcl-2, and Survivin (Figures 3(a) and 3(b)). We found that GSK-3*β* or LiCl only had no significant effect on the expression of these proteins (although LiCl reduced Bax expression, there was no statistical significance), and IL-1*β* increased Bax expression and inhibited Bcl-2 and Survivin expression. At the same time, the cointervention with GSK-3*β* enhanced these trends, while LiCl reversed them. Meanwhile, the expression of caspase 9, cleaved caspase 9, caspase 3, and cleaved caspase 3 were also detected, and the results were consistent (Figures 3(c) and 3(d)). In addition, the flow cytometric analysis (Figures 3(e) and 3(f)) and TUNEL staining (Figure 3(g)) were performed to assess the number of apoptotic cells. IL-1*β* markedly increased the cell apoptosis compared to the control group, and the addition of GSK-3*β* exacerbated this effect, while LiCl reversed it.

### 3.4. GSK-3*β* Regulates the NF-*κ*B and Wnt/*β*-Catenin Signaling Pathways in IL-1*β*-Induced Inflammation

To explore the possible molecular mechanism, we investigated the NF-*κ*B and Wnt/*β*-catenin signaling pathways in BMSCs. In this study, IL-1*β* significantly stimulated the phosphorylation of IKK*α*/*β*, I*κ*B*α*, and NF-*κ*B p65, which was enhanced by the addition of GSK-3*β*. Interestingly, only NF-*κ*B phosphorylation was reversed by LiCl (Figures 4(a) and 4(b)). In addition, we found that the phosphorylation of GSK-3*β* was significantly increased in the LiCl+IL-1*β* group. And compared with the IL-1 group, the phosphorylation of *β*-catenin was increased in the GSK-3*β*+IL-1*β* group while decreased in the LiCl+IL-1*β* group (Figures 5(a)–5(d)).

### 3.5. GSK-3*β* Mediates the Cross-Reaction between NF-*κ*B and *β*-Catenin in the Nucleus

Furthermore, the expression of NF-*κ*B and *β*-catenin in the cytosol and nucleus were detected. IL-1*β* increased NF-*κ*B expression in the nucleus, and GSK-3*β* enhanced this trend, while LiCl and SN50 reversed it (Figures 4(c)–4(f)). Meanwhile, IL-1*β* decreased *β*-catenin expression in the nucleus, and GSK-3*β* enhanced this trend, while LiCl reversed it (Figures 5(e) and 5(f)). Newly, after cointervention with SN50, a specific inhibitor of NF-*κ*B translocation, *β*-catenin expression in the nucleus was significantly increased (Figures 5(g) and 5(h)). Meanwhile, immunofluorescence was performed (Figure 6). The results showed that GSK-3*β* promoted the IL-1*β*-induced nuclear translocation of NF-*κ*B p65, while LiCl and SN50 decreased it. And in the IL-1*β* group and the GSK-3*β*+IL-1*β* group, the green fluorescence signal (*β*-catenin) could be clearly observed in the cytoplasm, but there was almost no signal in the nucleus. However, in the LiCl+IL-1*β* group, the SN50+IL-1*β* group and the SN50+GSK-3*β*+IL-1*β* group, the green fluorescence signal in cytoplasm was significantly reduced, and only slight signal was observed in the nucleus.

## 4. Discussions

Bone marrow mesenchymal stem cells can be induced to differentiate into chondrocytes under certain conditions, which has potential application value in the treatment of cartilage diseases [17]. In agreement with previous studies, we showed that IL-1*β* suppresses the chondrogenesis ability and cartilage matrix synthesis ability of BMSCs and also induces BMSCs apoptosis during the process of chondrogenesis [13, 17–20]. It has been shown that GSK-3*β* is extensively involved in the regulation of glucose metabolism, cell proliferation, differentiation, migration, and apoptosis [21–25] and plays a key role in chondrogenic differentiation [26]. In this study, we found GSK-3*β* exacerbated the effects detected by IL-1*β* stimulation, which could be reversed by LiCl.

We further investigated the molecular mechanisms of GSK-3*β* affecting chondroblast differentiation and apoptosis in an inflammatory microenvironment. Previous studies have confirmed the involvement of GSK-3*β* in the regulation of NF-*κ*B activation [7, 8]. Therefore, the regulation of NF-*κ*B signaling pathway by GSK-3*β* was first detected. It was found that GSK-3*β* could activate NF-*κ*B signaling pathway, and only NF-*κ*B phosphorylation was reversed by LiCl. Similarly, Schwabe and Brenner reported that treatment of TNF-*α*-stimulated cells with LiCl resulted in a decrease of the NF-*κ*B-dependent gene transcription, but did not affect I*κ*B*α* degradation or IKK activity [27]. Meanwhile, in our study, GSK-3*β* promoted nuclear translocation of NF-*κ*B p65, which was attenuated by inhibition of GSK-3*β* activity (LiCl) or NF-*κ*B translocation inhibitor (SN50).

A large number of studies have shown that the Wnt/*β*-catenin signaling pathway plays an essential role in regulating cell proliferation and differentiation [28–31], and GSK-3*β* is the crucial regulator of the Wnt/*β*-catenin signaling pathway [30]. Next, we examined the regulation of GSK-3*β* on Wnt/*β*-catenin signaling pathway. As expected, GSK-3*β* upregulated the phosphorylation of *β*-catenin, while LiCl inhibited the activity of GSK-3*β* and thus downregulated the phosphorylation of *β*-catenin. Furthermore, we detected the expression of *β*-catenin in the nucleus and found that it was significantly decreased after GSK-3*β* stimulation. This may be due to the phosphorylation of *β*-catenin leading to its degradation, thereby reducing the nuclear translocation [32]. Importantly, the expression of *β*-catenin in the nucleus was increased when nuclear translocation of NF-*κ*B p65 was specifically inhibited by SN50, suggesting a cross-reaction between NF-*κ*B and *β*-catenin in the nucleus.

In summary, our study confirmed the role of GSK-3*β* in chondrogenic differentiation of BMSCs in IL 1*β*-induced inflammatory microenvironment. Additionally, our research provides a new insight into the molecular mechanisms that GSK-3*β* regulates the chondrogenesis via NF-*κ*B and Wnt/*β*-catenin signaling pathways and mediates the cross-reaction between NF-*κ*B and *β*-catenin in the nucleus (Figure 7).

## Figures and Tables

**Figure 1:** Chondrogenic differentiation of BMSCs in an IL-1*β*-induced inflammatory microenvironment. (a) and (b) Representative images and intensity quantification of Alcian blue staining. (c) The GAG content in the culture medium. The expression level of Sox9, Collagen 2a and Aggrecan were detected by qRT-PCR (d) and western blotting (e) and (f). All results are expressed as the mean ± SD (*n* = 3). NS: not significant, ^∗^*P* < 0.05 and ^∗∗^*P* < 0.01. Bar = 800 *μ*m.

**Figure 2:** GSK-3*β* disrupts metabolic balance of IL-1*β*-impaired BMSCs. (a) Representative immunofluorescence images of collagen 2a. (b) The GAG content in the culture medium. (c) The expression level of Sox9, C and Aggrecan were detected by qRT-PCR (c) and western blotting (d) and (e). All results are expressed as the mean ± SD (*n* = 3). NS: not significant and ^∗^*P* < 0.05. Bar = 1000 *μ*m.

**Figure 3:** GSK-3*β* promotes apoptosis of IL-1*β*-impaired BMSCs. (a)-(d) The expression level of caspase 9, cleaved caspase 9, caspase 3, cleaved caspase 3, Bax, Bcl-2, and Survivin were detected by western blotting. Flow cytometric analysis (e) and (f) and TUNEL staining (g) were performed to assess the number of apoptotic cells. All results are expressed as the mean ± SD (*n* = 3). NS: not significant, ^∗^*P* < 0.05. Bar = 800 *μ*m.

**Figure 4:** GSK-3*β* regulates the NF-*κ*B signaling pathway in IL-1*β*-induced inflammation. Phosphorylation and/or total expression of IKK*β*, IKK*α*/*β*, I*κ*B*α*, and NF-*κ*B p65 (a) and (b) were detected by western blotting. Visualization and quantification of the expression of cytoplasmic (c) and (d) and nuclear (e) and (f) NF-*κ*B p65. All results are expressed as the mean ± SD (*n* = 3). NS: not significant, ^∗^*P* < 0.05, and ^∗∗^*P* < 0.01.

**Figure 5:** GSK-3*β* regulates the Wnt/*β*-catenin signaling pathway in IL-1*β*-induced inflammation. Phosphorylation and total expression of GSK-3*β* (a) and (b) and *β*-catenin (c) and (d) were detected by western blotting. (e)-(h) visualization and quantification of the expression of nuclear *β*-catenin. All results are expressed as the mean ± SD (*n* = 3). NS: not significant, ^∗^*P* < 0.05, and ^∗∗^*P* < 0.01.

**Figure 6:** GSK-3*β* mediates the cross-reaction between NF-*κ*B and *β*-catenin in the nucleus. Immunofluorescence was used to observe the distribution of NF-*κ*B p65 (red) and *β*-catenin (green). The nuclei were DAPI-stained (blue). Three independently repeated experiments were performed, and a representative image is shown. Bar = 100 *μ*m.

**Figure 7:** Schematic diagram of the mechanisms. GSK-3*β* regulates the chondrogenesis via NF-*κ*B signaling and Wnt/*β*-catenin signaling and possibly mediates the cross-reaction between NF-*κ*B and *β*-catenin in the nucleus.

**Table 1:** The information of primers.

Gene	Sequences	
*Sox9*	Forward	5′-GTGGGAGCGACAACTTTACC-3′
	Reverse	5′-GCGAGCACTTAGCAGAGGC-3′
*Collagen 2a*	Forward	5′-CACCCAGAGTGGAAGAGCG-3′
	Reverse	5′-TCAGTGGACAGTAGACGGAGGA-3′
*Aggrecan*	Forward	5′-CAAACAGCAGAAACAGCCAAGT-3′
	Reverse	5′-GAAGGCATAAGCATGTGAAAGTG-3′
*GAPDH*	Forward	5′-AACGACCCCTTCATTGACCTC-3′
	Reverse	5′-CCTTGACTGTGCCGTTGAACT-3′

## Data Availability

The original contributions presented in the study are included in the article; further inquiries can be directed to the corresponding author.
